# Machine Algorithm for Heartbeat Monitoring and Arrhythmia Detection Based on ECG Systems

**DOI:** 10.1155/2021/7677568

**Published:** 2021-12-30

**Authors:** Ahmed I. Taloba, Rayan Alanazi, Osama R. Shahin, Ahmed Elhadad, Amr Abozeid, Rasha M. Abd El-Aziz

**Affiliations:** Department of Computer Science, College of Science and Arts in Qurayyat, Jouf University, Sakakah, Saudi Arabia

## Abstract

Cardiac arrhythmia is an illness in which a heartbeat is erratic, either too slow or too rapid. It happens as a result of faulty electrical impulses that coordinate the heartbeats. Sudden cardiac death can occur as a result of certain serious arrhythmia disorders. As a result, the primary goal of electrocardiogram (ECG) investigation is to reliably perceive arrhythmias as life-threatening to provide a suitable therapy and save lives. ECG signals are waveforms that denote the electrical movement of the human heart (P, QRS, and T). The duration, structure, and distances between various peaks of each waveform are utilized to identify heart problems. The signals' autoregressive (AR) analysis is then used to obtain a specific selection of signal features, the parameters of the AR signal model. Groups of retrieved AR characteristics for three various ECG kinds are cleanly separated in the training dataset, providing high connection classification and heart problem diagnosis to each ECG signal within the training dataset. A new technique based on two-event-related moving averages (TERMAs) and fractional Fourier transform (FFT) algorithms is suggested to better evaluate ECG signals. This study could help researchers examine the current state-of-the-art approaches employed in the detection of arrhythmia situations. The characteristic of our suggested machine learning approach is cross-database training and testing with improved characteristics.

## 1. Introduction

The electrocardiogram (ECG) is used to measure the electrical activity of the heart. In many circumstances, analyzing the ECG signal might provide an understanding of life-threatening cardiac disorders. These researchers are typically disturbed with recognizing and diagnosing different types of diseases such as arrhythmias, which are described as an enlarged rate of heart or a disruption in the rate of a normal person [1]. Irregularities in heart rhythm can be caused by a variety of factors, including illness drugs, an aging heart, or metabolic issues. Sustained ventricular arrhythmia is among the most dangerous arrhythmias, which is frequently caused by the destroyed heart muscle. Cardiovascular disease (CVD) is the important cause of mortality worldwide, accounting for around 31% of all deaths worldwide. The heart is a cone-shaped organ system that pumps at regular intervals to deliver blood to the internal tissues [2]. A heart attack happens due to an obstruction in the coronary arteries, which deliver blood and oxygen to the heart.

According to the World Health Organization, CVDs constitute the major public health problem worldwide. Various initiatives and policies are applied in more diverse communities in recent years and offer tools, tactics, and other resources to minimize occurrences of the first and recurring cardiovascular actions. In the end, the ECG has been developed to be the most widely employed biosignal for the early diagnosis of CVDs [3]. The ECG is a schematic illustration of the heart electrical activity that is utilized to diagnose different heart illnesses and irregularities. For more than 70 years, doctors have used ECG electrical signals to diagnose heart problems, include arrhythmia and heart attack.  Figure 1 shows an ECG signal that comprises complex P, QRS, and T waves. A U-wave could also be present. Many heart illnesses can be identified by studying the fluctuations of these waves. ECG technologies are both harmless and affordable. However, noise and other variables were known as artifacts that will cause jumps in the ECG signals [4]. These artifacts can include patient physical movements, electrode motion on the body, and external electrical interference.

To overcome the shortcomings of the aforementioned algorithms, an approach is suggested based on the TERMA fusion and fractional Fourier transform (FFT) that can yield superior results. Moving averages (MA) are useful in recognizing signals that comprise detailed occurrences, and TERMA is mostly used in economics to distinguish the various measures in trading [3]. As a result, these averages can be applied to ECG data that comprise events including T waves and P, QRS complex. These waves continue by themselves after a given amount of time. Because of the substantial variability in the T waves and P, QRS complex, time-frequency studies are also significant. This explains that moving averaging and time-frequency studies can be used to detect these waves. Furthermore, it was demonstrated that the suggested approach in this work outperforms the existing techniques significantly.

An autoregressive (AR) signal model order as *j*, AR(*j*), was used to simulate a minimum number of consecutive ECG signals. The model parameters obtained are employed as ECG signal characteristics and categorized using several common algorithms for classification. The results show that these features are well separated in the retrieved space and give accurate classification and identification of various cardiac diseases [5]. Moreover, sets of retrieved AR values were used to identify specific individuals from recorded ECG signals. Initial findings show that this method has the potential to be used in various biometric situations. The rest of the research discusses the scheme that was used to retrieve and categorize those characteristics and some outcomes for detection of arrhythmia and information of patient tasks [6].

The next task is to determine and characterize any CVD in an ECG signal. The classification process consists of two steps: extraction of features and classifier model selection. Using a database of MIT-BIH arrhythmia, many scholars have focused on the ECG signals classification. Previous research used a variety of preprocessing models, methods of feature extraction, and classifiers, some of which are covered in this research [7]. Discrete wavelet transform (DWT) is utilized to retrieve characteristics like the R peak and RR interval, and multilayer perceptron (MLP) has been utilized in the methods of classification. Similarly, the R peak region and RR interval are identified using db4 DWT; a feedforward neural network (FFNN) is developed with backpropagation to identify ECG signals. In classification, various classifiers were utilized, including support vector machines (SVM), neural networks, AdaBoost, and Naive Bayes [8].

## 2. Literature Review

The study in [9] evaluated irregular heartbeats, including heart failure, cardiac arrhythmias, and sinus rhythms. The electrocardiogram (ECG) is an important and widely used tool for detecting and classifying cardiac infractions. A heart ECG signal analyzes the heart's electrical activity and produces waveforms that can be used to diagnose cardiac abnormalities. As a result of this research, it is possible to classify arrhythmias with greater accuracy and a shorter SVM classifier with discrete wavelet transform (DWT) is the machine learning technique used in this study. From the MIT-BIH and BIDMC databases, seventy-three percent of the composed signals are divided into training and testing sets, with 70 : 30. DWT was used to extract a total of 190 features. Due to its flexibility to alter the window size based on frequency, DWT as a solution SVM classifier was used to classify the retrieved characteristics. For analysis, the findings used a testing set, and to visualize the final results, we used a model that has a 95.92 percent performance accuracy.

According to [10], heart-related illnesses (CVDs) have been responsible for a large number of deaths worldwide over the previous few decades, making them the world's leading cause of mortality. In recent years, many researchers have used a variety of machine learning algorithms to help the medical industry and healthcare providers diagnose heart-related problems. In conclusion, this study provides an overview of numerous models that focus upon these methods and methodologies. Naive Bayes, random forest (RF), k-nearest neighbor (KNN), decision trees (DT), support vector machines (SVM), and ensemble models are popular models, particularly among researchers.

In [11], to diagnose cardiac disease, the clinical and pathological data were combined in a sophisticated way. As a result of this complexity, clinical practitioners and researchers are very interested in developing a method for predicting cardiac disease that is efficient and an algorithm for guessing heart disease status depending on the clinical information is presented in this research. There are three steps to this strategy. In the beginning, choose 13 significant clinical variables, such as age and gender, type of chest pain, treetops and levels of cholesterol, fasting sugar in the blood, resting ECG, maximum rate of heart, and exercise-induced angina, old peak, and slop. To detect cardiac disease based on these clinical parameters, an algorithm based on artificial neural networks (ANN) is created. Approximately 80% of the predictions are right on target. As the last step, a user-friendly heart disease prediction system (HDPS) was developed. As a result of methods, a patient's heart condition can be accurately forecasted. As a result of this work, the HDPS system was developed, which is a revolutionary technology that may be employed in this method.

In [12], it was reported that mortality and morbidity from heart disease (HD) are on the rise in modern society. As a vital yet difficult task that must be completed precisely and efficiently, medical diagnosis automation would be extremely beneficial. There is a shortage of doctors in many parts of the world because not all doctors are equally adept in every subspecialty. In addition to enhancing medical treatment, an automated medical diagnosis system would also reduce the cost. In this research, a coactive neuro-fuzzy inference system (CANFIS) was employed to build a new technique for preventing heart illness. The proposed CANFIS for new diagnostic analysis combines an autonomous neural network system with a descriptive fuzzy-based method. Focusing on its training efficiency and accuracy rate, the proposed CANFIS algorithm is found to have significant ability in detecting cardiac disease.

The study in [13] presents a hybrid approach for optimally classifying cardiac arrhythmias and selecting their properties. The Genetic Method was utilized to optimally pick the characteristics in the suggested model, and the Decision Tree (DT) algorithm was utilized to extract the feature to organize and build the system. The planned method is utilized to categorize information into normal and pathologic categories, a 16-class arrhythmias collection. This can employ the UCI arrhythmia database, as well as selectivity, sensitivity, accuracy, and mean Sen-Spec parameters, to evaluate the effectiveness of the projected scheme to that of similar approaches. The suggested method's effectiveness in both two-class and 16-class modes greatly enhances the accuracy, sensibility, average sensitivity, and specificity metrics when compared to similar approaches. In terms of accuracy, sensitivity, and the mean Sen-Spec parameters, our approach achieved values of 86.96 percent, 88.88 percent, and 86.55 percent for the two-class model and 78.76 percent, 76.36 percent, and 78.69 percent for the 16-class model classification. The values listed above are the highest for the UCI arrhythmia database.

## 3. Methodology

The ECG categorization system developed in this article may be divided into four major stages, as shown in Figure 2. The following are the stages:

- Preprocessing ECG
- Detection of QRS and segmentation signal
- Extraction of parameter
- Extracted parameter classification and clustering

### 3.1. ECG Preprocessing

The preprocessing objective stage is to increase an overall ECG quality signal so that it can be analyzed and examined more accurately. The reduction of baseline deviations and the other patterns in a raw signal produced by the power line intrusions and the artifacts was the first stage in the ECG analysis process [14]. Background drift is an unnecessary minimum-frequency movement in ECG that can affect with analysis of the signal, resulting in incorrect and misleading clinical interpretation. Its spectrum content is typically much below 1 Hz, but higher frequencies may be present during intensive exercise.

Filtering is among the most popular ways for removing excessive noise and baseline drift from ECG readings. In the past, both FIR and IIR filter types were effectively used for this task, with lower and higher rates of cutoff in the 0.8 Hz and 40 Hz ranges, respectively. A cutoff frequency greater than 0.8 Hz has been documented to alter the waveform of ECG significantly, and it should be evaded. Bandpass filtering is utilized in this work to minimize and eliminate the noise disturbance that usually appears in ECG readings. The bandpass ECG filter has a lower cutoff frequency of 5 Hz and a higher cutoff wavelength of 40 Hz.

### 3.2. Detection of QRS

The QRS complex was the single greatest critical element of the ECG signal. For such a QRS complex, the start and delay of the QRS complex, as well as the P and T waveforms, are all defined. Most QRS recognition algorithms are built mainly on a filtering step trailed by the averaging based on a threshold value [15]. This threshold is being used to differentiate between the background and the QRS complex and is based on the ECG signal's top position. Other techniques based on machine learning include the method of P-spectrum, a powerful way of detecting periodicity derived from data discontinuity.

### 3.3. Extraction of the Parameter

At the next level of the system, AR modeling of the two or more consecutive ECG beats using the discrete variant of an AR signal model of order *j*, AR(*j*), is used after an individual heartbeat detection for each ECG signal. Each dataset's order *j* is determined by examining the variance of forecast errors as a function of basic functions *j*. Modeling two consecutive ECG beats identified using the filter bank method briefly mentioned in the preceding section yielded good results in this study [16]. The estimated model's coefficients are subsequently employed as classification signal characteristics in the design and system period. A signal sequence as *k*(*v*) will be described by the AR model in the following equation:

(1) $$\begin{array}{c} k\left(v\right)=x_{1}k\left(v-1\right)+x_{2}k\left(v-2\right)+x_{j}k\left(v-j\right)+\varepsilon \left(v\right). \end{array}$$

The model coefficients, commonly defined as the parameters of autoregressive, utilized in the classiﬁcation model are *x*_*f*_(*f*=1,2,…, *j*) and *ε*(*v*) is a white noise sequence, technology process with a zero mean, and variance *σ*^2^. In equation (2), the calculated autoregressive model is now regarded as a p-point predictions filter, only with actual output *k*(*v*) predicted from the preceding (*j*  −  1) AR processes target value.

(2) $$\begin{array}{c} \hat{j}\left(v\right)=\overset{j}{\underset{i=1}{\sum }}\hat{x_{f}}j\left(v-i\right), \end{array}$$

where $\hat{x_{f}}\left(f=1,2,\ldots ,j\right)$ characterize the assessed limits of the AR design.

### 3.4. Classification

The collected ECG signal characteristics were classified and recognized using various classification techniques. The multidimensional matrices carrying the calculated autoregressive parameters for every beat of the recorded ECG signal are a characteristic of this work. The k-nearest neighbor method is among the most commonly used approaches in bioinformatics and other fields due to its simplicity, although attention must be given while picking the model of order *k* as appropriate dimension measures. To the next stage of this study, the electrocardiography identifying patient characteristics was addressed and evaluated using linear (LDA) and quadratic (QDA) discriminant analysis classifiers employed in a different bioinformatics application.

### 3.5. Heartbeat Classifier

An echo state network (ESN) is used to create the suggested heartbeat classifier. It divides the analyzed electrocardiogram records' heart rates into two groups depending on morphological features: VEB+ and SVEB+. Normal (*N*) and supraventricular ectopic (*S* or SVEB) heartbeats were both classified as SVEB+. In contrast to VEB + heart rate, which has a ventricular source or aberrant morphology, those heart rates have a regular morphological characteristic and a supraventricular source. Ventricular ectopic beats (*V* or VEB) and fusion beats were included in the VEB + category (*F*).

Figure 3 depicts the complete procedure in schematic form. There is a clear distinction between the two phases:

- Stage 1: feature extraction, filtering, heartbeat segmentation, and heartbeat detection are all part of the first phase of ECG recorded analysis. In this approach, we integrate morphological and time pauses among heart rates.
- Stage 2: classification between SVEB+ and VEB + classes, to execute this classifying assignment, we utilize an ensemble of ESNs with ring topology. Further in the article, we go over the classification technique in phase two in greater depth, as shown in Table 1.

### 3.6. Feature Extraction and ECG Processor

Minor preprocessing of the original ECG recordings is required to achieve arrhythmia categorization. The basic methods are included in the analysis of ECG records in this framework.

#### 3.6.1. ECG Filtering

To adjust the foundation and eliminate undesirable high frequencies noises, every ECG recordings are processed in a bandwidth *ν* (Hz)  ∈ [0.5,  35]. With conventional technique, a Butterworth high-pass filter (with a cutoff frequency of *ν*_*c*_= 0.5 Hz) and a 12th-order limited impulse response filter (35 Hz, at 3 dB point) were utilized.

#### 3.6.2. Resampling of ECG Signals

ECG transmissions were analyzed at a monitoring frequency of 260 Hz. Utilizing the PhysioToolkit application programme, the AHA dataset (260 Hz) is kept at its normal recording frequency, while the MIT-BIH AR dataset (350 Hz) is normalized to 260 Hz.

#### 3.6.3. Computation of the RR Interval

The RR interval is measured as the period among succeeding heart rates. The duration comparison of heartbeat *i* and the preceding heartbeat (*i*−1) is represented by the RR interval linked with heartbeat *i*, RR(*i*)

#### 3.6.4. Heartbeat Detection

Annotated coordinates offered by datasets were employed to estimate the placement of heart rates. The annotating position in the MIT-BIHAR database is at the highest of the QRS complex's localized edges. The identification of beats is outside the focus of this research. There have also been reports of extremely effective automatic beat recognition systems.

#### 3.6.5. Normalization of Segmented Heartbeats

Every segmented heart rate is normalized among [1, 1]. This scalability technique yields a signal that is unaffected by the frequency of the initial ECG recordings.

#### 3.6.6. Heartbeat Segmentation

Every database's indicated position is used to segment the ECG signals. The segmented heart rates are 250 milliseconds long (65 samples per second at 250 Hz) and are centered on the annotated place.

Every heart rate is characterized by a collection of properties once the ECG recordings have been processed. Because we want to construct a rapid and real-time heartbeat classification, one of the key objectives of selecting parameters in this system is to prevent difficult characteristics with a large computing expense. As a result, we concentrate on straightforward methods for extracting characteristics. In our example, we display it with the actual waveform of every heartbeat between the heart rate points. Every beat's actual information was provided by an equivalent number of samples from every side of the beat identification position. Every pulse is displayed as a *d* − dimensional vector at the conclusion of the preprocessing and extraction of features phase, with three characteristics related to the RR intervals and 65 morphological features that are basically a sampling of the ECG waveform around the point indicated for every heart rate. The categorization technique takes this *d* − dimensional vector (*d* = 62) as inputs.

### 3.7. Waveform of ECG

ECG patterns are traces of the heart's electrical system and play an important role in the diagnosis method for analyzing physical health. A typical ECG trace is comprised of a P wave, QRS complex, and *T* wave during every ventricular contraction [17]. Arrhythmias are abnormal heartbeats that arise when the usual pattern of electrical impulses in the heart is disrupted. Arrhythmias can happen in both the lower and upper heart chambers, but ventricular arrhythmia will be experienced.

As previously stated, artifacts and noise in signals must be eliminated to identify P, QRS, and T waves. To identify P, QRS complex, and T waveforms, the traditional wavelet transform-based filtering technique is utilized to eliminate noise and artifacts. To improve detection accuracy, TERMA and FFT are combined machine learning methods that were utilized to identify the ECG signals and evaluate if there is any CVD. The next subsections go over the specific duties in further depth.

### 3.8. Signal Filtering

The ECG signals were nonstationary, which means that resonance frequency varies over a period of time. Also, the noise and objects contaminating the ECG signal were nonlinear, with a time-dependent probability density. Time localization is not possible with traditional Fourier transform techniques, but it is possible with DWT. As a result, DWT is more capable of dealing with nonstationary signals [18]. The first step is to use DWT to eliminate the average drift. To do so, first, compute the wavelet's core frequency, *R*_*c*_ (also known as the *F*_*c*_ factor), which ranges from 0 to 1 based on the signal's resemblance to the chosen waveform.

Daubechies-4 (db4) has the greatest *R*_*c*_ factor, equal to 0.7, for ECG signals. Then, at each level, the pseudofrequency, *R*_*a*_, is determined using the following equation:

(3) $$\begin{array}{c} R_{a}=\frac{R_{c}R_{s}}{2^{a}}, \end{array}$$

where *a* and *R*_*s*_ are the ECG signal's gauge and selection frequency, respectively. The majority of the baseline drift occurs at 0.5Hz. The scales equivalent to various pseudofrequencies will be easily computed using (3) for the MIT-BIH Fs = 360. Up to scale 9, which corresponds to *R*_*a*_  = 0.5, should be decomposed. As a result, the db4 wavelet divides the ECG signal into approximation and detailed coefficients up to scale 9. To find a baseline signal drift-free, the estimated coefficients related to the drift baseline were eliminated, and the signal was rebuilt using IDWT.

### 3.9. Fusion Algorithm to Detect R Peaks

At the R peak in ECG signal, there was greatest change in the frequency. The time localization can be compromised when using the Fourier transform of the ECG data. FFT should be used to the noise-free information in this stage to transform it in the time-frequency domain. The FFT operation includes chirp multiplying, chirp inversion, and another chirp multiplication, as shown in the arrangements [19]. Rotation of the information with a higher value is comparable to getting closer to the transmitter resonant frequency; however, moving that with a reduced amount is equal to moving away from the signal's resonant frequency, which is equivalent to getting closer to the signal's temporal domain. Time localization is crucial when it comes to R peak detection. Using the hit-and-trial techniques, it was discovered that the parameter of *α*= 0.01 boosts R peaks properly and makes them difficult to recognize. By squaring each sample after applying FFT, then the R peak was increased more. Following the enhancement, the two MAs depending on event and cycle are determined:

(4) $$\begin{array}{c} {\text{MA}}_{\text{event}}\left(n\right)=\frac{1}{U_{1}}\overset{j}{\underset{i=-j}{\sum }}a\left(n+i\right),\\ {\text{MA}}_{\text{cycle}}\left(n\right)=\frac{1}{U_{2}}\overset{c}{\underset{i=-c}{\sum }}a\left(n+c\right). \end{array}$$

MA is represented as moving average, *U*_1_  is determined by the length of the QRS complex, and *U*_2_ is determined by the length of the heartbeat. The augmented signal's mean (*μ*) is determined and increased by factor (*β*); the optimum parameter value was determined using the hit-and-miss approach. The output value was applied to MA_cyclic_ producing threshold values and is represented by *γ*=*βμ*. The MA_event_ values were compared to the relevant threshold values. One is assigned if MA_event_(*n*) is greater than the nth criterion. A new vector is created if zero is not provided. This produces a stream of nonuniform distribution rectangular pulses.

Finally, illustrated in Figure 4, the pulses with widths equal to *U*_1_ are the blocks that include the anticipated event. The R peak value for every block is the high value in the accompanying improved signal. This procedure is described in depth. After applying the suggested technique, the R peaks were accurately recognized.

### 3.10. Detection of P and T Peak Using Fusion Algorithm

TERMA employs a complex threshold to identify P and T peaks. Using a reduced threshold, we were able to minimize the algorithm's overall processing complexity. The R peaks are removed in the first phase of the algorithm, allowing the P and T peaks to be more noticeable. In the noise-free signal, 30 samples (0.083 s) were well earlier than the R peak and the 60 samples (0.166 s); then, the R peak value was set to 0 [20]. For any CVD, the probability of the P and T waves in the specified interval was practically nil. The signal was replaced in a time-frequency plane using the FFT to boost the P and T peaks after the QRS interval was removed. Blocks of interest were formed in the same way as in the following step, as illustrated in Figure 5, utilizing two moving axes:

(5) $$\begin{array}{c} {\text{MA}}_{\text{peak}}\left(n\right)=\frac{1}{U_{3}}\overset{d}{\underset{i=-d}{\sum }}a\left(n+d\right),\\ {\text{MA}}_{\text{wave}}\left(n\right)=\frac{1}{U_{4}}\overset{e}{\underset{i=-e}{\sum }}a\left(n+e\right). \end{array}$$

W3 is determined by the frequency of the P wave, W4 is determined by the QT interval, *d*=*U*_3_ − 1/2, and *e*=*U*_4_ − 1/2 W421. The P wave duration in a fit individual will be (100 ± 20) ms; then, the QT interval will be (400 ± 40) ms. Instead of using a standard size window to identify P waves, a minimum window is used to account for unique characteristics of the arrhythmias. The measurements were just the values of the next moving average, as opposed to the R peak detection. One is assigned if the initial average was higher than the comparable next moving average. A new vector is created if the zero is not get assigned. This produces a stream of nonuniform rectangular impulses. Finally, to separate the created blocks from blocks containing P and T peaks, a threshold depending on the intervals of PR, RR, and RT was used. The highest power of the block is referenced as the P peak if the gap is between the highest benefits of the block and the nearest R peak on the specified PR interval. If the difference only between the appropriate dosage of the component and the closest R peak is below a prescribed RT period, the highest values of the blocks were referred to as as T peak.

### 3.11. Machine Learning Supervised Algorithms

The categorization of ECG signals is a crucial and difficult endeavor. It will deliver a great deal of information about a patient's CVDs without the need for cardiology. Only a specialist is needed to connect the inquiries, and also machine learning-based system will detect a patient's CVDs immediately [21]. This method can quickly identify people that require rapid medical intervention. The MLP and SVM supervised learning techniques are employed for the classification in this study and explained temporarily in the subcategories below.

### 3.12. SVM Classifier

In regression and classification issues, the SVM algorithm can be employed. Information is displayed in the space of l-dimensional in SVM, with l being the variety of attributes. Following the graph of the information, classification is carried out by locating a hyperplane, distinguishing between several classes [22]. The hyperplane is optimized via maximization of the margin. The hyperplane that is nearest to the nearest information points between the other hyperplanes is picked. The ratio that indicates the issue is fixed by the SVM:

(6) $$\begin{array}{c} \max_{x\geq 0}\left(\overset{j}{\underset{g=1}{\sum }}\alpha_{g}-\frac{1}{2}\overset{j}{\underset{g,h=1}{\sum }}\alpha_{g}\alpha_{h}p_{g}p_{h}I\left(A_{g},A_{h}\right)\right), \end{array}$$

subject to

(7) $$\begin{array}{c} \overset{j}{\underset{g=1}{\sum }}\alpha_{g}p_{g}=0,\\ \alpha_{g}\leq W,\;g=1,2,\ldots ,j, \end{array}$$

where *α*_*g*_ ≥ 0 are the Lagrangian multipliers, *W* is denoted as constant, and *K*(*X*, *X*_1_) is a kernel function, where *A*_*g*_, *A*_*h*_ are the input features, *p*_*g*_, *p*_*h*_ are class labels. The Gaussian radial basis function is a widely popular kernel.

(8) $$\begin{array}{c} K\;\left(X,\;X_{1}\right)=\exp-\frac{{\left\|X,\;X_{1}\right\|}^{2}}{2\sigma^{2}}. \end{array}$$

In higher-dimensional environments, the number of sizes exceeds the number of models and the SVM is particularly successful.

### 3.13. Multilayer Perceptron Classifier

Artificial neural network (ANN) methods identify zones using an approach that mimics human brain functions like comprehending, learning, problem-solving, and decision-making. Three layers make to the ANN model. The input image is the initial layer, and the number of neurons in this sheet are determined by input parameters [23]. The output layer is the final layer, with the hidden neurons representing the number of the output classes. The hidden layers exist among the hidden layer and the output layer. MLP is a feedforward neural ANN subclass used during this study.

## 4. Results and Discussion

This segment is divided into four sections that are focused on recognition of arrhythmias, detection of the peak, cross-database training and testing, and classification, respectively.

### 4.1. Recognition of Arrhythmias

To assess the effectiveness of the proposed scheme, an ECG set of results containing three different types of ECG signals has been used. The dataset contained normal ECG signals (NR) from Politecnico of Milano VCG/ECG Data on Young Normal Subject, arrhythmia (AR) from the MIT-BIH Arrhythmia Database, and ventricular arrhythmia (VAR) again from MIT-BIH Malignant Ventricular Arrhythmia Database. Every kind was represented by 20 half-hour records of two-channel outpatient ECG data, although the testing just took minutes for each person. After the beat recognition and signal separation steps, AR parameters are produced for each extracted group of beats. The frequency of beats in each band and also the number of AR parameters collected for each team could all have an effect on the performance of the classifying program. The effective classification was achieved for 1–5 beats in the band and 2–4 AR variables. This shows the performance of the two beats per set with AR order *p* values of two and three in this study.  Figure 6 depicts the error values for different AR-type orders for both preprocessed and raw ECG signals. However, more difficult procedures are normally employed to decide the model order; the modeling error plot's breakpoint (“knee”) is being used to choose a model or models.

The “knee point” position in Figure 6 is of lesser risk, which is determined to be adequate for such heavily processed ECG signals with an AR basis function of 2 or 3. Making extra orders has no discernible effect on modeling error or classification process accuracy. For processing ECG signals, the discontinuity in this chart is immediately evident (2 or 3); however, the same spot in the raw ECG plot is more difficult to identify. It is also worth noting that the modeling error for the processed signal is substantially smaller than the error modeling acquired when modeling the raw ECG data.

Furthermore, the variation of recovered variables should really be observed, as evidenced by the size of related feature clouds in AI feature space. When comparing the variations of the information clouds to distinguish between the two arrhythmias, the dimensionality of the data cloud associated with daily ECG signals is comparatively small, also with ventricular arrhythmia cloud containing the maximum variation and dispersion of image features.

### 4.2. ECG Detection of Peaks

The P, R, and T peaks are discovered in the initial portion of the simulation using our proposed FFT-based approach, and the suggested algorithm is validated across all 48 records in the MIT-BIH. This research makes use of Lead II (MLII) data. Because our approach is not affected by the magnitude of the waveforms, any following information will be helpful for the detection of the peak. Furthermore, the performance can be evaluated using various metrics described in the literature, including positive predictivity, failure rate, and sensitivity as follows:

(9) $$\begin{array}{c} \text{positive predictivity }\left(+\text{PP}\right)=\frac{\text{TP}}{\text{FP}+\text{TP}},\\ \text{failure rate }\left(\text{Frr}\right)=\frac{\text{TP}+\text{FP}}{\text{TP}},\\ \text{sensitivity }\left(\text{ST}\right)=\frac{\text{TP}}{\text{FN}+\text{TP}}, \end{array}$$

where TP means true positive, FN represents false negative considered as marked peaks not discovered by the system, and FP represents false positive as the peaks identified by method but not simply present. If a peak is discovered within a 30 ms of the annotation peak, it is well defined as TP. This evaluated TP, FN, and FPs to measure the algorithm's efficiency.

### 4.3. CVD Classification

In the next portion of the experiment, the ECG signals are categorized according to their CVDs. For all simulations, 70% of the selected features were used to train a machine learning model, while 30% was kept for test results. As a result, various features were retrieved from the waveforms for classification. The collected features were then sent into the SVM and MLP classifications, which were used to categorize the input ECG signals as regular, PVC, APC, LBBB, RBBB, and PACE heartbeats. The following performance measures were utilized to evaluate the proposed classifier's effectiveness to that of the current ones:

(10) $$\begin{array}{c} \text{overall accuracy}=\frac{\text{TN}+\text{TP}}{\text{TN}+\text{TP}+\text{FN}+\text{FP}},\\ \text{recall}=\frac{\text{TP}}{\text{FP}+\text{TP}},\\ \text{precision}=\frac{\text{TP}}{\text{FN}+\text{TP}},\\ f_{1}-\text{score}=2.\;\frac{\text{recall}\times \text{precision}}{\text{recall}+\text{precision}}, \end{array}$$

where TN stands for true negative, which means that the person has a CVD and the classifier indicates that the individual is not normal.

### 4.4. Testing and Training Database

The MLP classifiers are trained using the MIT-BIH arrhythmia collection and subsequently evaluated on the INCART22 and SPH23 databases in St. Petersburg to classify the normal, RBBB, and PVC heartbeats. The sample rates in each of the three datasets varied. As a result, for convenience, all of the data were resized to a frequency of 128 Hz. There was no requirement for preprocessing because the data retrieved from these sources were already free of baseline drift and noise. Age, gender, PR, and RT intervals are among the objective truth. The trained model's accuracy rate on the IN CART and SPH databases was 99.85 percent and 68 percent, respectively. The suggested approach had been unable to identify inverted, biphasic negative-positive, and biphasic positive-negative T peaks that may be observed in RBBB and PVC; the classification was unable to accurately categorize the RBBB and PVC heartbeats. As a result, its average classification accuracy suffers. There is a disadvantage to cross-database analysis. In both training and testing, illness features were normalized and the normal patient characteristics were not normalized. When applying normalization to all the testing and training data, the classifier's exactness suffers even further. This illness is unreal and requires more research.

## 5. Conclusion

A method for automatically classifying ECG data into three groups has been presented in arrhythmia and ventricular arrhythmia. To detect the R, P, and T peaks, a fusion technique based on FFT and TERMA was presented. To denoise data, conventional wavelet transform methods were used; however, the introduction of FFT in the TERMA techniques dramatically enhanced peak detection accuracy. The proposed peak identification performs the role marginally better than the TERMA algorithm in detecting the R peak but much improved in detecting the P and T peaks in the MIT-BIH arrhythmia collection. Following the preprocessing processes, AR modeling is utilized to extract the AR parameters that are used to categorize every portion of the ECG signal into each of three potential categories. Selected features and AR characteristics for sets of the two beats are highly divided in the feature space and effectively categorized, suggesting that excellent classification accuracy may be anticipated in the suggested system's effective implications. Furthermore, unlike the TERMA method, the effectiveness was not affected by CVDs. Following peak identification, the results are utilized to determine the PR and RT periods as characteristics of two ECG signals for classification constructed a classifier for the cross-database testing and training.

## Figures and Tables

**Figure 1:** Normal ECG morphology.

**Figure 2:** Proposed ECG main blocks.

**Figure 3:** Fully automatic heartbeat classifier.

**Figure 4:** Detection of the R peaks: a block of interests is generated.

**Figure 5:** Detection of the P and T peaks and then interest block is generated.

**Figure 6:** AR model for order selection.

**Table 1:** The training (DS1) and testing (DS2) sets' heartbeat class distributions.

Database	SVEB + class		VEB + class	
	*N*	*S*	*V*	*F*
AHA (DS1)	159,688		15,086	293
AHA (DS2)	157,998		15,866	448
MIT-BIH AR	45,794	954	3,796	425
MIT-BIH AR	44,189	1,945	3,217	392

## Data Availability

The data used to support the findings of this study are included within the article.
